# Different Data Mining Approaches Based Medical Text Data

**DOI:** 10.1155/2021/1285167

**Published:** 2021-12-06

**Authors:** Wenke Xiao, Lijia Jing, Yaxin Xu, Shichao Zheng, Yanxiong Gan, Chuanbiao Wen

**Affiliations:** ^1^School of Medical Information Engineering, Chengdu University of Traditional Chinese Medicine, Chengdu 611137, China; ^2^School of Pharmacy, Chengdu University of Traditional Chinese Medicine, Chengdu 611137, China

## Abstract

The amount of medical text data is increasing dramatically. Medical text data record the progress of medicine and imply a large amount of medical knowledge. As a natural language, they are characterized by semistructured, high-dimensional, high data volume semantics and cannot participate in arithmetic operations. Therefore, how to extract useful knowledge or information from the total available data is very important task. Using various techniques of data mining can extract valuable knowledge or information from data. In the current study, we reviewed different approaches to apply for medical text data mining. The advantages and shortcomings for each technique compared to different processes of medical text data were analyzed. We also explored the applications of algorithms for providing insights to the users and enabling them to use the resources for the specific challenges in medical text data. Further, the main challenges in medical text data mining were discussed. Findings of this paper are benefit for helping the researchers to choose the reasonable techniques for mining medical text data and presenting the main challenges to them in medical text data mining.

## 1. Introduction

The era of big data is coming with the mass of data growing at an incredible rate. The concept of big data for the first time was put forward in the 11th EMC World conference in 2011, which refers to large-scale datasets that cannot be captured, managed, or processed by common software tools. With the arrival of big data age, the amount of medical text data is increasing dramatically. Analyzing this immense amount of medical text data to extract the valuable knowledge or information is useful for decision support, prevention, diagnosis, and treatment in medical world [1]. However, analyzing the huge amount of multidimensional or raw data is very complicated and time-consuming task. Data mining has capabilities for this matter.

Data mining is a methodology for discovering the novel, valuable, and useful information, knowledge, or hidden pattern from enormous datasets by using various statistical approaches. Data mining is with many advantages in contrast to the traditional model for transforming data to knowledge with some manual analysis and interpretation. Data mining approaches are quicker, favorable, time-saving, and objective. Summarizing various data mining approaches in medical text data for clinical applications is essential for health management and medical research.

This paper is organized in four sections.  Section 2 presents the concepts of medical text data.  Section 3 includes data mining approaches and its applications in medical text data analysis.  Section 4 concludes this paper and presents the future works.

## 2. Medical Text Data

The diversity of big data is inseparable from the abundance of data sources. Medical big data including experimental data, clinical data, and medical imaging data are increasing with the rapid development of medicine. Medical big data are the application of big data in the medical field after the data related to human health and medicine have been stored, searched, shared, analyzed, and presented in innovative ways [2]. Medical text data are an important part of medical big data which are described in natural language, cannot participate in an arithmetic operation, and are characterized by semistructured, high-dimensional, high data volume semantics [3]. They cannot be well applied in research owing to no fixed writing format and being highly professional [4]. Medical text data contain clinical data, medical record data, medical literature data, etc., and this type of data records the progress of medicine and implies a large amount of medical knowledge. However, utilizing human power to extract the facts of relationships between entities from a vast amount of medical text requires time-consuming efforts. With the development of data mining technology, data mining technology used for medical text to discover the relationships in medical text becomes the hot topic. Medical text data mining is able to assist the discovery of medical information. In the COVID-19 research field, medical text mining can help decision-makers to control the crown outbreak by gathering and collating scientific basic data and scientific research literature related to the new crown virus, predicting the susceptible population to new crown pneumonia, virus variability, and potential therapeutic drugs [5–8].

## 3. Medical Text Data Mining

Data mining was defined in the “First section of the 1995 International Conference on Knowledge Discovery and Data Mining,” which has been widely used in disease auxiliary diagnosis, drug development, hospital information system, and genetic medicine to facilitate the medical knowledge discovery [9–12]. Data mining used to process medical text data can be divided into four steps: data collection, data processing, data analysis, and data evaluation and interpretation. This study summarized the algorithms and tools for medical text data based on the four steps of data mining.

### 3.1. Data Preparation

Medical text data include electronic medical records, medical images, medical record parameters, laboratory results, and pharmaceutical antiquities according to the different data sources. The different data were selected based on the data mining task and stored in the database for further processing.

### 3.2. Data Processing

The quality of data will affect the efficiency and accuracy of data mining and the effectiveness of the final pattern. The raw medical text data contain a large amount of fuzzy, incomplete, noisy, and redundant information. Taking medical records as an example, the traditional paper-based medical records have many shortcomings, such as nonstandard terms, difficult to form clinical decision-making support, scattered information distribution, and so on. After the emergence of electronic medical records, the medical records data are gradually standardized [13]. However, the electronic medical records still as natural language are difficult for data mining. Therefore, it is necessary to clean up and filter the data to ensure data consistency and certainty by removing missing, incorrect, noisy, and inconsistent or no quality data.

Missing values in medical text data are usually handled by deletion and interpolation. Deletion is the easiest method to handle, but some useful information is lost. Interpolation is a method that assigns reasonable substitution values to missing values through a specific algorithm. At present, many algorithms have emerged in the process of data processing. Multiple imputation, regression algorithm, and *K*-nearest neighbors are often used to supplement missing values in medical text data. The detail algorithm information is shown in Table 1. In order to further understand the semantic relationships of medical texts, researchers have used natural language processing (NLP) techniques to perform entity naming, relationship extraction, and text classification operations on medical text data with good results [19].

#### 3.2.1. Natural Language Processing

Natural Language Processing (NLP) as a subfield of artificial intelligence is mainly used for Chinese word segmentation, part-of-speech tagging, parsing, natural language generation, text categorization, information retrieval, information extraction, text-proofing, question answering, machine translation, automatic summarization, and textual entailment with the advantage of the fast process and lasting effect. It affirms positive motivation without negative influence, which can effectively stimulate potential, keep learning, keep growing, and keep developing [20].

In medical text processing, NLP is often used for information extraction and entity naming including word segmentation, sentence segmentation, syntactic analysis, grammatical analysis, and pragmatic analysis. The schematic of natural language processing is shown in Figure 1. Kou et al. [21] used NLP tools to extract important disease-related concepts from clinical notes, form a multichannel processing method, and improve data extraction ability. Jonnagaddala et al. [22] proposed a hybrid NLP model to identify Framingham heart failure signs and symptoms from clinical notes and electronic health record (EHR). Trivedi et al. [23] designed an interactive NLP tool to extract information from clinical texts, which can serve clinicians well after evaluation. Datta et al. [24] evaluated the NLP technology to extract cancer information from EHR, summarized the implementation functions of each framework, and found many repetitive parts in different NLP frameworks resulting in a certain waste of resources. The possibility of diversified medical text data will also bring the transformation of medical data analysis mode and decision support mode. Roberts and Demner-Fushman [25] manually annotated tags on 468 electronic medical records to generate a corpus, which provided corpus support for medical data mining. The development of NLP technology greatly reduces the difficulty of manual data processing in data mining. Shikhar Vashishth et al. [26] used semantic type filtering to improve the performance connectivity of medical entities across all toolkits and datasets, which provided a new semantic type prediction module for the biomedical NLP pipeline. Topaz et al. [27] used an NLP-based classification system, support vector machine (SVM), recurrent neural network (RNN), and other machine learning methods to identify diabetic patients from clinical records and reduce the manual workload in medical text data mining.

### 3.3. Data Analysis

Data analysis is applying data mining methods for extracting interesting patterns. The model establishment is essential for knowledge discovery in data analysis. According to the characteristics of the data, modeling and analysis are performed. After the initial test, the model is parametrically adjusted. The advantages and disadvantages of different models are analyzed to choose the final optimal model. Data analysis methods for medical text data include clustering, classification, association rules, and regression on the goal. The detail information of methods is shown in Table 2.

#### 3.3.1. Artificial Neural Network

Artificial Neural Network (ANN) is a nonlinear prediction model that is learned by training, which has the advantages of accurate classification, self-learning, associative memory, and high speed searching for the optimal solution and good stability in data mining. ANN mainly consists of three parts: input layer, hidden layer, and output layer [40]. The input layer is responsible for receiving external information and data. The hidden layer is responsible for processing information and constantly adjusting the connection properties between neurons, such as weights and feedback, while the output layer is responsible for outputting the calculated results. ANN is different from traditional artificial intelligence and information processing technology, which overcomes the drawbacks of traditional artificial intelligence based on logical symbols in processing intuitive and unstructured information, and has the characteristics of self-adaption, self-organizing, and real-time learning. It can complete data classification, feature mining, and other mining tasks. Medical text data contain massive amounts of patient health records, vital signs, and other data. ANN can analyze the conditions of patients' rehabilitation, find the law of patient data, predict the patient's condition or rehabilitation, and help to discover medical knowledge [41].

There are several ANN mining techniques that are used for medical text data, such as backpropagation and factorization machine-supported neural network (FNN). The information on ANN mining techniques is shown in Table 3.

*(1) ANN Core Algorithm: BP Algorithm*. Backpropagation (BP) algorithm, as the classical algorithm of the ANN, widely used for medical text data. BP algorithm is developed on the basis of single-layer neural network. It uses reverse propagation to adjust the weights and construct multilayer network, so that the system can continue to learn. BP is a multilayered feed-forward network and its propagation is forward. Compared with recurrent neural network algorithms, error spreads reversely makes it faster and more powerful for high-throughput microarray or sequencing data modeling [45].

BP algorithm training data is mainly divided into the following two stages:

(1) Forward propagation process: the actual output values of each computer unit are implicitly processed layer by layer from the input layer
(2) Backpropagation process: when the output value does not reach the expected value, the difference between the actual output and the expected output is calculated recursively, and the weight is adjusted according to the difference. The total error is defined as
  (1) $$\begin{array}{c} E=\sum_{k=1}^{m}E_{k}=\sum_{k=1}^{m}\sum_{t=1}^{q}\frac{{\left(y_{t}^{k}-c_{t}^{k}\right)}^{2}}{2}. \end{array}$$
*m* is the total number of samples. *K* is the sample data order. *T* is the unit serial number. *y*_*t*_^*k*^ is the desired output. *c*_*t*_^*k*^ is the actual output.

In clinics, the judgment of disease is often determined by the integration of multidimensional data. In the establishment of disease prediction models, BP algorithms can not only effectively classify complex data but also have good multifunctional mapping. The relationship between data and disease can be found in the process of repeated iteration [46].

*(2) Application Examples*. Adaptive learning based on ANN can find the law of medical development from the massive medical text data and assist the discovery of medical knowledge. Heckerling et al. [47] combined a neural network and genetic algorithm to predict the prognosis of patients with urinary tract infections (as shown in Figure 2). In this study, nine indexes (eg, frequent micturition, dysuria, etc.) from 212 women with urinary tract infections were used as predictor variables for training. The relationship between symptoms and urinalysis input data and urine culture output data was determined using ANN. The predicted results were accurate.

Miotto et al. [48] derived a general-purpose patient representation from aggregated EHRs based on ANN that facilitates clinical predictive modeling given the patient status. Armstrong et al. [49] used ANN to analyze 240 microcalcifications in 220 cases of mammography. Data mining results can accurately predict whether the microcalcification in the early stage of suspected breast cancer is benign or malignant.

#### 3.3.2. Naive Bayes

Naive Bayes (NB) is a classification counting method based on the Bayes theory [50]. The conditional independence hypothesis of the NB classification algorithm assumes that the attribute values are independent of each other and the positions are independent of each other [51]. Attribute values are independent of each other, which means there is no dependence between terms. The position independence hypothesis means that the position of the term in the document has no effect on the calculation of probability. However, conditional dependence exists among terms in medical texts, and the location of terms in documents contributes differently to classification [52]. But medical text existence conditions depend on the relationship between a middle term and the term in the document; the location of the contribution to the classification is different. These two independent assumptions lead to the poor effect of NB estimation. However, NB has been widely used in medical texts because it plays an effective role in classification decision-making.

*(1) Core Algorithm: NBC4D*. Naive Bayes classifier for continuous variables using a novel method (NBC4D) is a new algorithm based on NB. It classifies continuous variables into Naive Bayes classes, replaces traditional distribution techniques with alternative distribution techniques, and improves classification accuracy by selecting appropriate distribution techniques [53]. The implementation of the NBC4D algorithm is mainly divided into five steps:

1. Gaussian Distribution: $\;f\left(x,\;\mu ,\;\sigma \right)=1/\sigma \sqrt{2\pi }e^{-{\left(x-\mu \right)}^{2}/2\sigma^{2}}$
2. Exponential Distribution*:f*(*x*)=1/*αe*^−*x*/*θ*^
3. Kernel Density Estimation: *f*(*x*)=1/*nh*∑_*i*=1_^*n*^*K*(*x* − *x*_*i*_/*h*)
4. Rayleigh Distribution:  *f*(*x*,  *α*,  *θ*)=*x*/*αe*^−*x*^2^/2*θ*^
5. NBC4D Method: find the product of the probability (possibility) of each attribute of a given specific class and the probability of a specific class to improve the accuracy

*x* is the input value, *μ* is the mean value, *σ*_*2*_ is the variance, *α* is the parameter that represents the average value *(μ)*, *θ* represents the standard deviation (*σ*), *K* is the kernel function of Gaussian function, and *h* is the smoothing parameter.

*(2) Application Examples.* Behrouz Ehsani Moghaddam et al. [54] adopted electronic medical records (EMRs) extracted from the Canadian primary care sentinel surveillance network, used the Naive Bayes algorithm to classify disease features, and found that Naive Bayes classifier was an effective algorithm to help physicians diagnose Hunter syndrome and optimize patient management (as shown in Figure 3). In order to predict angiographic outcomes, Golpour et al. [55] used the NB algorithm to process the hospital medical records and assessment scale and found that the NB model with three variables had the best performance and could well support physician decision-making.

#### 3.3.3. Decision Tree

The decision tree is a tree structure, in which each nonleaf node represents a test on a feature attribute, each branch represents the output of the feature attribute on a certain value domain, and each leaf node stores a category [56]. The process of using a decision tree to make a decision is to start from the root node, then test the corresponding characteristic attributes of the items to be classified, select the output branch according to its value until it reaches the leaf node, and finally take the category stored in the leaf node as the decision result [57]. The advantages of decision tree learning algorithms include good interpretability induction, various types of data processing (categorical and numerical data), white-box modeling, sound robust performance for noise, and large dataset processing. Medical text data is complex [58]. For instance, electronic medical record data include not only disease characteristics but also patient age, gender, and other characteristic data. Since the construction of decision tree starts from a single node, the training data set is divided into several subsets according to the attributes of the decision node, so the decision tree algorithm can deal with the data types and general attributes at the same time, which has certain advantages for the complexity of medical text data processing [59]. The construction of a decision tree is mainly divided into two steps: classification attribute selection and number pruning. The common algorithm is C4.5 [60].

*(1) Core algorithm: C4.5*. Several decision tree algorithms are proposed such as ID3 and C4.5. The famous ID3 algorithm proposed by Quinlan in 1986 has the advantages of clear theory, simple method, and strong learning ability. The disadvantage is that it is only effective for small datasets and sensitive to noise. When the training data set increases, the decision tree may change accordingly. When selecting test attributes, the decision tree tends to select attributes with more values. In 1993, Quinlan proposed the C4.5 algorithm based on the ID3 algorithm [61]. Compared with ID3, C4.5 overcomes the shortages of selecting more attributes in information attribute selection, prunes the tree construction process, and processes incomplete data. And it uses the gain ratio as the selection standard of each node attribute in the decision tree [62]. In particular, its extension which is called S-C4.5-SMOTE and can not only overcome the problem of data distortion but also improve overall system performance. Its mechanism aims to effectively reduce the amount of data without distortion by maintaining the balance of datasets and technical smoothness.

The processing formula is as follows:

(2) $$\begin{array}{c} \text{Information entropy}:H\left(x\right)=-\overset{n}{\underset{i=1}{\sum }}p\left(x_{i}\right)\log_{2}\;p\left(x_{i}\right),\\ \text{Split information}\left(A,S\right)=-\overset{c}{\underset{i=1}{\sum }}\frac{\left|Si\right|}{\left|S\right|}\log\;2\frac{\left|Si\right|}{\left|S\right|},\\ \text{Gain ratio }\left(A,S\right)=\frac{\text{Gain}\left(S,A\right)}{\text{Split information}\left(S,A\right)}. \end{array}$$

*n* is the classification number. *p(x*_*i*_) represents the proportion of sample *x*_*i*_*. A* is used as the feature of dividing data set *S*. (|*Si*|/|*S*|) is the proportion of the number of samples in the total number of samples.

*(2) Application Examples*. The decision tree algorithms can construct specific decision trees for multiattribute datasets and get feasible results in relative time. It can be used as a good method for data classification in medical text data mining.

Byeon [63] used the C4.5 algorithm to develop a depression prediction model for Korean dementia caregivers based on a secondary analysis of the 2015 Korean Community Health Survey (KCHS) survey results. And the effective prediction rate was 70%. The overall research idea is shown in Figure 4.

Wei et al. [64] selected the reports from the Chinese spontaneous report database from 2010 to 2011 and used a decision tree to calculate the classification of adverse drug reactions (ADR) signals. Tao Zheng et al. [65] adopted a decision tree algorithm to construct a basic data framework. 300 data were randomly selected from the EHR of 23281 diabetic patients to classify the type of diabetes. The performance of the framework was good and the classification accuracy was as high as 98%.

However, decision tree algorithms are difficult to deal with missing values in data. And there are many missing values in medical text data, due to the high complexity of data. Therefore, when various types of data are inconsistent, the decision tree algorithms will produce information deviation, and the correct results cannot be obtained.

#### 3.3.4. Association Rules

Association rules are often sought for very large datasets, whose efficient algorithms are highly valued. They are used to discover the correlations from large amounts of data and reflect the dependent or related knowledge between events and other events [66]. Medical text data contains a large number of association data, such as the association between symptoms and diseases and the relationship between drugs and diseases. Mining medical text data using an association rule algorithm is conducive to discovering the potential links in medical text data and promoting the development of medicine. Association rules are expressions like *X* ≥ *Y*. There are two key expressions in the transaction database:

1. Support{*X*≥*Y*}. The ratio of the number of transactions with *X* and *Y* to all transactions
2. Confidence{*X*≥*Y*}. The ratio of the number of transactions with *X* and *Y* to the number of transactions with *X*

Given a transaction data set, mining association rules is to generate association rules whose support and trust are greater than the minimum support and minimum confidence given by users, respectively.

*(1) Core Algorithm: Apriori*. The apriori algorithm is the earliest and the most classic algorithm. The iterative search method is used to find the relationship between items in the database layer by layer. The process consists of connection (class matrix operation) and pruning (removing unnecessary intermediate results). In this algorithm, the concept of item set is the set of items. A set containing *K* items is a set of *K* items. Item set frequency is the number of transactions that contain an item set. If an item set satisfies the minimum support, it is called a frequent item set.

Apriori algorithm is divided into two steps to find the largest item set:

1. Count the occurrence frequency of an element item set, and find out the data set which is not less than the minimum support to form a one-dimensional maximum item set
2. Loop until no maximum item set is generated

*(2) Application Examples*. Association rules are usually a data mining approach used to explore and interpret large transactional datasets to identify unique patterns and rules. They are often used to predict the correlation between index data and diseases. Exarchos et al. [67] proposed an automation method based on association rules, used an association rule algorithm to classify and model electrocardiographic (ECG) data, and monitored ischemic beats in ECG for a long time. In this study, the specific application process of association rules is shown in Figure 5.

Hrovat et al. [68] combined association rule mining, which was designed for mining large transaction datasets, with model-based recursive partitioning to predict temporal trends (e.g., behavioral patterns) for subgroups of patients based on discharge summaries. In the correlation analysis between adverse drug reaction events and drug treatment, Chen et al. [69] used the apriori algorithm to explore the relationship between adverse events and drug treatment in patients with non-small-cell lung cancer, showing a promising method to reveal the risk factors of adverse events in the process of cancer treatment. In the association between drugs and diseases, Lu et al. [70] used the apriori algorithm to find herbal combinations for the treatment of uremic pruritus from Chinese herb bath therapy and explore the core drugs.

### 3.4. Model Evaluation

Classifications generated by data mining models through test sets are not necessarily optimal, which can lead to the error of test set classification. In order to get a perfect data model, it is very important to evaluate the model. Receiver operating characteristic (ROC) curve and area under the curve (AUC) are common evaluation methods in medical text data mining.

The ROC curve has a *y*-axis of TPR (sensitivity, also called recall rate) and an *x*-axis of FPR (1-specificity). The higher the TPR, the smaller the FPR, and the higher the efficiency of the model. AUC is defined as the area under the ROC curve, that is, AUC is the integral of ROC, and the value of the area is less than 1. We randomly select a positive sample and a negative sample. The probability that the classifier determines that the positive sample value is higher than the negative sample is the AUC value. Pourhoseing Holi et al. [71] used the AUC method to evaluate the prognosis model of rectal cancer patients and found that the prediction accuracy of random forest (RF) and BN models was high.

## 4. Discussion

Data mining is useful for medical text data to extract novel and usable information or knowledge. This paper reviewed several research works which are done for mining medical text data based on four steps. It is beneficial for helping the researchers to choose reasonable approaches for mining medical text data. However, some difficulties in medical text data mining are also considered.

First, the lack of a publicly available annotation database affects the development of data mining to a certain extent, due to differences in medical information records and descriptions among countries. Its information components are highly heterogeneous and the data quality is not uniform. Ultimately, it brings about a key obstacle that makes annotation bottleneck existing in medical text data [72]. At present, the international standards include ICD (International Classification of Diseases), SNOMED CT (The Systematized Nomenclature of Human and Veterinary Medicine Clinical Terms), CPT (Current Procedural Terminology), DRG (Diagnosis-Related Groups), LOINC (Logical Observation Identifiers Names and Codes), Mesh (Medical Subject Headings), MDDB (Main Drug Database), and UMLS (Unified Medical Language System). There are few corpora in the field of medical text. In recent 10 years, natural language has undergone a truly revolutionary paradigm shift. More new technologies have been applied to the extraction of natural language information. Many scholars have established a corpus for a certain disease. However, there is a close relationship between medical entities. A single corpus cannot cut the data accurately, and it is easy to omit keyword information.

Second, text records of different countries have different opinions. For example, Ayurvedic medicine, traditional Arab Islamic medicine, and traditional Malay medicine from India, the Middle East, and Malaysia have problems such as inconsistent treatment description, complex treatment methods, and difficulty in statistical analysis, leading to great difficulty in medical data mining [73]. At the same time, the information construction of traditional medicine is insufficient. For example, the traditional North American indigenous medical literature mainly involves clinical efficacy evaluation and disease application, which is complicated in recording methods, leading to difficulty of data mining [74]. Chinese medical texts have the particularity of language. Unlike English expressions, Chinese words are not separated from each other, which increases the difficulty of data analysis. In terms of semantics, Chinese medical texts have problems such as existential polysemy, synonym, the ambiguity of expression, complex relationship, and lack of clear correlation. Building a standard database based on these data is very difficult, which requires very advanced and complex algorithms.

In addition, the electronic medical record contains personal privacy information. Sometimes, the clinical electronic medical record data will inevitably be used in medical text data mining. Therefore, the protection of patient privacy data is also an issue that needs to be paid attention to in data mining.

In future work, we will attempt to establish and popularize medical text data standards with the help of intelligent agents and construct publicly available annotation databases for the mining of medical text data.

## Figures and Tables

**Figure 1:** Schematic of natural language processing flow.

**Figure 2:** ANN algorithm analysis process.

**Figure 3:** NB algorithm analysis process.

**Figure 4:** C4.5 algorithm application flow.

**Figure 5:** Application process of association rules.

**Table 1:** The detailed algorithm information for missing values in medical text data.

Algorithm	Principle	Purpose
Multiple imputation [14, 15]	Estimate the value to be interpolated, and add different noises to form multiple groups of optional interpolation values; select the most appropriate interpolation value according to a certain selection basis.	Repeat the simulation to supplement the missing value
Expectation maximization [16]	Compute maximum likelihood estimates or posterior distributions with incomplete data.	Supplement missing values
*K*-nearest neighbors [17, 18]	Select its *K* closest neighbors according to a distance metric and estimate missing data with the corresponding mode or mean.	Estimate missing values with samples

**Table 2:** The information of analysis methods for medical text data.

Methods	Purpose	Algorithms	Advantages	Shortcomings
Clustering	Classify similar subjects in medical texts	*K*-means [28, 29]	1.Simple and fast 2. Scalability and efficiency	1. Large amount of data and time-consuming 2. More restrictions on use

Classification	Read medical text data for intention recognition	ANN [30, 31]	1. Solve complex mechanisms in text data 2. High degree of self-learning 3. Strong fault tolerance	1. Slow training 2. Many parameters and difficulty in adjusting parameters
		Decision tree [32, 33]	1. Handle continuous variables and missing values 2. Judge the importance of features	1. Overfitting 2. The result is unstable
		Naive bayes [34]	1. The learning process is easy 2. Good classification performance	Higher requirements for data independence

Association rules	Mine frequent items and corresponding association rules from massive medical text datasets	Apriori [35, 36]	Simple and easy to implement	Low efficiency and time-consuming
		FP-tree [37]	1. Reduce the number of database scans 2. Reduce the amount of memory space	High memory overhead
		FP-growth [38]	1. Improve data density structure 2. Avoid repeated scanning	Harder to achieve
Logistic Regression	Analyze how variables affect results	Logistic regression [39]	1.Visual understanding and interpretation 2. Very sensitive to outliers	1.Easy underfitting 2. Cannot handle a large number of multiclass features or variables

**Table 3:** The information of ANN mining techniques.

ANN mining techniques	Advantages	Shortcomings
Backpropagation [42]	1. Strong nonlinear mapping capability 2. Strong generalization ability 3. Strong fault tolerance	1. Local minimization 2. Slow convergence 3. Different structure choices
Radial basis function [43]	1. Fast learning speed 2. Easy to solve text data classification problems	Complex structure
FNN [44]	1.Reduce feature engineering 2. Improve FM learning ability	Limited modeling capability

## Data Availability

No data were used to support this study.

## Abbreviations

EMC: The U.S.A EMC company
NLP: Natural language processing
ANN: Artificial neural network
BP: Backpropagation
ROC: Receiver operating characteristic
TPR: True positive rate
FPR: False positive rate
AUC: Area under the curve
RF: Random forest
BN: Bayesian network
EHR: Electronic health record
ICD: International classification of diseases
SNOMED CT: The systematized nomenclature of human and veterinary medicine clinical terms
CPT: Current procedural terminology
DRG: Diagnosis-related groups
Mesh: Medical subject headings
LOINC: Logical observation identifiers names and codes
UMLS: Unified medical language system
MDDB: Main drug database
SVM: Support vector machine
RNN: Recurrent neural network
ID3: Iterative Dichotomiser 3
KCHS: Korean community health survey
ADR: Adverse drug reactions
ECG: electrocardiographic
FNN: Factorization machine-supported neural network.
